# The Clinical Nursing Pathway on Prevention of Catheter Slippage with Intensive Care Unit Patients: A Systematic Review and Meta-Analysis

**DOI:** 10.1155/2022/1144888

**Published:** 2022-09-13

**Authors:** Huanhuan Huang, Shanzhao Yu, Jufang Zheng

**Affiliations:** Department of Intensive Care Unit, Affiliated Hospital of Shaoxing University, Shaoxing, Zhejiang 312000, China

## Abstract

**Objective:**

To evaluate the prevention effect of the clinical nursing pathway (CNP) of catheter slippage with intensive care unit (ICU) patients.

**Methods:**

Primary databases were electronically searched from the inception up to June 25, 2021. Randomized clinical trials of CNP versus routine nursing for prevention of catheter slippage with ICU patients were included. The risk of bias was assessed using the Cochrane risk of bias tool and the quality of included studies using the Jadad rating scale. A meta-analysis was conducted using the Cochrane collaboration's RevMan5.3 software.

**Results:**

Eight studies met the inclusion criteria. The findings of the meta-analysis revealed that the comparison of CNP and routine nursing was applied in ICU patients, the catheter slippage incidence rate odds ratio (OR) was 0.11, with 95% confidence interval (CI) (0.05, 0.24), and the difference was statistically significant (*P* < 0.00001). The catheter infection rate OR was 0.15, with 95% CI (0.06, 0.37), and the difference was statistically significant (*P* < 0.0001). The nursing satisfaction OR was 14.06, with 95% CI (5.71, 34.63), and the difference was statistically significant (*P* < 0.00001).

**Conclusion:**

Compared with routine nursing, the application of CNP in ICU patients can effectively reduce the incidence of catheter slippage, reduce the infection rate of the catheter, and improve the nursing satisfaction.

## 1. Introduction

The intensive care unit (ICU) is a hospital department that treats critically ill patients. Patients admitted to the ICU are often serious with various diseases or conditions, and most patients have catheters left in the body during treatment [1, 2]. Some patients may have catheter slippage during the treatment process, affecting the quality of the patient's prognosis [3]. Catheter slippage, also known as an unplanned extubation, is the accidental shedding of the catheter or the removal of the catheter without the consent of the medical staff, including the extubation caused by incorrect operation of the medical staff [4, 5]. Catheter care is an essential component of critical patient care, and the quality of care provided during the treatment is associated with the overall quality of prognosis of hospitalized patients [6, 7]. Currently, the focus of ICU care work is concentrated on how to improve the quality of care for ICU patients and limit the occurrence of catheter slippage [8, 9]. Indwelling catheter patients are now implementing the clinical nursing pathway (CNP) to prevent catheter slippage. Based on CNP, the nurse can rate the ICU patients to determine the catheter slippage risk. Patients with high-risk levels are identified as high-risk groups, and the corresponding nursing measures are determined according to the different risk levels. Many research has been conducted to compare the preventative impact of CNP to routine nursing [10, 11]. However, there is no systematic review reporting the effect of CNP on the prevention of catheter slippage in ICU patients. As a result, we comprehensively evaluated the effect of CNP on prevention of catheter slippage in ICU patients compared with routine nursing.

## 2. Materials and Methods

### 2.1. Literature Search Strategy

Major Chinese and English databases were searched, including the Chinese National Knowledge Infrastructure (https://www.cnki.net/; CNKI), the Wanfang database (https://www.wanfangdata.com.cn/), the Chongqing VIP information (https://www.cqvip.com/; CQVIP), Cochrane Central Register of Controlled Trials (https://www.cochrane.org/; CENTRAL), and PUBMED (https://www.ncbi.nlm.nih.gov/pubmed). The search period was from the inception to June 25, 2021.

The search terms included “clinical nursing pathway” and “ICU” or “intensive care unit” and “catheter slippage” or “unplanned extubation.”

### 2.2. Inclusion and Exclusion Criteria

Inclusion criteria included the following: the eligibility criteria complied with PICOS (participant, intervention, comparison, outcome, and study design) principles; the study subject is a nursing method of ICU patients (*P*); experimental group intervention includes combining CNP (*I*); control group intervention is routine nursing (*C*); the primary outcome is catheter slippage incidence rate (*O*); and the study is a randomized controlled trial (RCT) (*S*).

Exclusion criteria included the following: experimental group or control group includes other nursing method interventions and studies with incomplete primary outcome measures.

### 2.3. Quality Assessment and Data Extraction

The included studies were evaluated for quality based on the Cochrane risk of bias tool from the Cochrane Handbook V.5.1.0., and according to the predeveloped quality assessment form, including the risk bias evaluation on the included studies of random sequence generation, allocation concealment, blindness, data completeness, and selective reporting [12]. The included studies were evaluated for methodological quality using the Jadad rating scale, including randomization (0–2 points), blinding (0–2 points), and dropouts and withdrawals (0–1 points), less than 3 points as low-quality study, and more than 3 points as high-quality study [13]. The data of the included literature was then extracted, including the authors, year of publication, number of cases, interventions, and outcome indicators. For incomplete data, the information was further clarified by contacting the authors. Quality assessment and data extraction were performed by two independent researchers. In case of disagreement, a decision was made through discussion or by a third researcher.

### 2.4. Statistical Analyses

The included studies were subjected to a systematic review, and meta-analyses of the included studies were conducted using the RevMan 5.3 software. First, the heterogeneity among the included studies was evaluated; in the case of heterogeneity (*P* < 0.1, *I*^2^ ≥50%), a subgroup analysis or a random effects model was used. However, if there was no heterogeneity (*P* > 0.1, *I*^2^ <50%), a fixed-effect model was used [14, 15]. Dichotomous data were expressed as 95% confidence interval (CI), odds ratio (OR), and continuous data were expressed as 95% CI mean difference (MD). Publication bias was assessed by a funnel plot for the included studies [16]. Statistical significance was indicated as *P* < 0.05.

## 3. Results

### 3.1. Literature Search Results

A total of 76 references were obtained by searching the above databases. Duplicates were excluded, the titles and abstracts of the literature were thoroughly read, and finally, ten relevant studies were left. According to the inclusion criteria and exclusion criteria, the full text was read carefully, and excluded one retrospective [17] and one nonrandomized study [18]. Finally, eight RCTs were included [10, 11, 19–24].  Figure 1 depicts the screening procedure and the outcomes of the literature search.

### 3.2. Basic Characteristics of the Included Studies

A total of eight RCTs were included [10, 11, 19–24]. All the included studies were conducted in China and were mostly single-centered studies. All included experimental groups in the study were combined CNP, and the control group was routine nursing.  Table 1 presents the basic characteristics of the included studies.

### 3.3. Methodological Quality of the Included Studies

Two studies used a table of random digits for methods of randomization [23, 24], the remaining studies were not explicitly introduced. None of the studies mentioned allocation concealment, none introduced blindness, and there were no selectively reported results. The result data were complete (Figures 2 and 3). Jadad score for each study (2 studies) [23, 24] had 2 points, and the remaining six studies had 1 point. The risk of bias and quality of included RCTs are presented in Table 2.

### 3.4. Outcome Indicators

All the eight studies [10, 11, 19–24] compared the catheter slippage incidence rate, three studies [10, 22, 23] compared the catheter infection rates, and five studies [10, 11, 22–24] compared nursing satisfaction. However, one study [24] compared depression scale scores, anxiety scale scores, extubation time, and length of stay (Table 3).

### 3.5. Meta-Analysis

#### 3.5.1. Catheter Slippage Incidence Rate

All eight studies [10, 11, 19–24] compared the catheter slippage incidence rate. The heterogeneity test showed *P*=1.00 and *I*^*2*^ = 0%, indicating that there was no heterogeneity among the included studies. A fixed effect model was then selected (the pooled OR = 0.11, 95% CI 0.05–0.24, and *P* < 0.00001). The difference in catheter slippage incidence rate was significant in the experimental group than in the control group (Figure 4).

#### 3.5.2. Catheter Infection Rate

Three studies [10, 22, 23] compared catheter infection rates. The heterogeneity test showed *P*=0.99 and *I*^*2*^ = 0%, indicating that there was no heterogeneity among the included studies. A fixed effect model was then selected (the pooled OR = 0.15, 95% CI 0.06–0.37, and *P* < 0.0001). The difference in the catheter infection rate was significant in the experimental group than in the control group (Figure 5).

#### 3.5.3. Nursing Satisfaction

Five studies [10, 11, 22–24] compared nursing satisfaction. The heterogeneity test showed *P*=0.98 and *I*^*2*^ = 0%, indicating that there was no heterogeneity among the included studies. A fixed effect model was then selected (the pooled OR = 14.06, 95% CI 5.71–34.63, and *P* < 0.00001). The difference in nursing satisfaction was significant in the experimental group than in the control group (Figure 6).

#### 3.5.4. Publication Bias

Publication bias was analyzed by funnel plots, using the catheter slippage incidence rate as an example, with OR value of each result as the horizontal coordinate and the SE (log [OR]) as the longitudinal coordinate. Funnel plots indicated inverted and symmetric funnel shapes, suggesting no significant publication bias. The funnel plot of the catheter slippage incidence rate is depicted in Figure 7.

## 4. Discussion

Critically ill patients in ICU generally require various catheters, including tracheal catheters, central venous catheters, gastric tubes, urinary catheters, surgical area drainage tubes, and others. However, in ICU, catheter slippage events occur frequently, affecting the quality of the prognosis of patients [25, 26]. Catheter slippage is mainly caused by the accidental shedding of the catheter, but there is also the phenomenon of unauthorized extubation by patients, including the catheter slippage caused by incorrect operation of medical personnel [27, 28]. The incidence of catheter slippage must be limited to ensure the quality treatment of critically ill patients, promote their physical rehabilitation, avoid and prevent the occurrence of infection, and build a harmonious doctor-patient relationship.

CNP may assist nurses in performing the nursing work with foresight and initiative, so that patients can fully understand their nursing goals and can participate in the nursing process of the treatment [29, 30]. The CNP is formulated based on the different standards of patients every day, which can standardize the diagnosis and treatment behavior, improve medical quality, shorten hospital stay, control medical costs, and improve doctor-patient communication, as well as patient satisfaction [31–33].

Eight RCTs were included in this study. The meta-analyses revealed that the catheter slippage incidence rate in the CNP experimental group was significantly lower than that in the routine nursing control group (*P* < 0.00001). Catheter infection rate and nursing satisfaction were found to be associated with catheter slippage; hence, reducing the catheter slippage rate may reduce the infection rate of catheters and improve nursing satisfaction. Therefore, meta-analyses of catheter infection rate and nursing satisfaction were performed. The catheter infection rate in the CNP experimental group was significantly lower than that in the routine nursing control group (*P* < 0.0001); the nursing satisfaction in the CNP experimental group was significantly higher than that in the routine nursing control group (*P* < 0.00001). Furthermore, a single study [24] showed that the CNP experimental group also performed better than the routine nursing control group with regard to the depression scale score, anxiety scale score, extubation time, and length of hospital stay.

Meta-analysis is a statistical method that comprehensively collects all relevant studies and strictly evaluates and analyzes them individually, and then quantitatively processes the data to draw comprehensive conclusions [34]. Currently, meta-analysis is widely used in clinical practice and the evidence-based level of the conclusion is relatively high [35]. There are limited studies on the systematic review and meta-analysis of clinical nursing. This study included RCTs comparing CNP and routine nursing. Three studies [10, 21, 22] showed no statistically significant difference in the catheter slippage incidence rate between CNP and routine nursing. Two studies [10, 11] revealed no statistically significant difference in nursing satisfaction between CNP and routine nursing. The meta-analysis also determined the advantages of the CNP in the incidence of catheter slippage and satisfaction with nursing.

There are certain limitations in this systematic review. The quality of the included studies is low, the statistical sample number is not estimated, and many studies do not have clear random methods and clear blind methods, affecting the accuracy of the conclusions. However, the study subjects were the clinical nursing of ICU patients, and to some extent, the random methods and blind method had less impact on the study, so that the related bias was small, and the funnel plot showed no obvious publication bias, so the conclusions of this meta-analysis are still of considerable significance. Despite the relatively low Jadad scores of the included studies, we carefully reviewed the literature to ensure that the findings are true and reliable. More high-quality RCTs are required to obtain the best evidence.

## 5. Conclusions

To summarize, the application of the CNP can effectively reduce the incidence of catheter slippage, reduce the catheter infection rate, and improve nursing satisfaction compared with the routine nursing in ICU patients. However, the overall quality of the included studies is low, and more high-quality RCTs are needed to obtain significant evidence further.

## Figures and Tables

**Figure 1:** Literature search flow diagram.

**Figure 2:** Risk of bias graph.

**Figure 3:** Risk of bias summary.

**Figure 4:** Forest plot of comparison: catheter slippage incidence rate.

**Figure 5:** Forest plot of comparison: catheter infection rate.

**Figure 6:** Forest plot of comparison: nursing satisfaction.

**Figure 7:** Funnel plot of catheter slippage incidence rate.

**Table 1:** Summary of the included RCTs.

First author (ref)	Study year	Country	Sample size (experimental/control)	Experimental	Control
Huang [19]	2012	China	160 (88/72)	CNP	Routine nursing
Chen [20]	2015	China	140 (66/74)	CNP	Routine nursing
Lao [21]	2015	China	120 (60/60)	CNP	Routine nursing
Yu [22]	2016	China	68 (34/34)	CNP	Routine nursing
Liu [23]	2017	China	176 (88/88)	CNP	Routine nursing
Yu [24]	2018	China	88 (44/44)	CNP	Routine nursing
Ye [10]	2018	China	56 (28/28)	CNP	Routine nursing
Zhang [11]	2020	China	92 (46/46)	CNP	Routine nursing

RCT: randomized controlled trial; CNP: clinical nursing pathway.

**Table 2:** The risk of bias and Jadad score for the included studies.

First author (ref)	Study year	Random sequence generation	Allocation concealment	Blinding of patient	Blinding of assessor	Incomplete outcome data	Selective reporting	Other bias	Jadad score
Huang [19]	2012	*U*	*U*	*U*	*U*	*L*	*L*	*L*	1
Chen [20]	2015	*U*	*U*	*U*	*U*	*L*	*L*	*L*	1
Lao [21]	2015	*U*	*U*	*U*	*U*	*L*	*L*	*L*	1
Yu [22]	2016	*U*	*U*	*U*	*U*	*L*	*L*	*L*	1
Liu [23]	2017	*L*	*U*	*U*	*U*	*L*	*L*	*L*	2
Yu [24]	2018	*L*	*U*	*U*	*U*	*L*	*L*	*L*	2
Ye [10]	2018	*U*	*U*	*U*	*U*	*L*	*L*	*L*	1
Zhang [11]	2020	*U*	*U*	*U*	*U*	*L*	*L*	*L*	1

*L*: low risk of bias, *H*: high risk of bias, and *U*: unclear risk of bias.

**Table 3:** Primary outcomes of the included studies.

First author (ref)	Study year	Primary outcomes	Primary results (effect size)
Huang [19]	2012	Catheter slippage incidence rate	OR, 0.11 [0.01, 0.89]

Chen [20]	2015	Catheter slippage incidence rate	OR, 0.12 [0.01, 0.96]

Lao [21]	2015	Catheter slippage incidence rate	OR, 0.24 [0.03, 2.19]

Yu [22]	2016	Catheter slippage incidence rate Catheter infection rate Nursing satisfaction	OR, 0.12 [0.01, 1.01] OR, 0.15 [0.03, 0.75] OR, 25.71 [1.43, 462.31]

Liu [23]	2017	Catheter slippage incidence rate Catheter infection rate Nursing satisfaction	OR, 0.10 [0.01, 0.81] OR, 0.13 [0.03, 0.61] OR, 13.48 [3.05, 59.51]

Yu [24]	2018	Catheter slippage incidence rate Nursing satisfaction Depression scale score Anxiety scale score Extubation time Length of stay	OR, 0.08 [0.01, 0.65] OR, 9.80 [2.07, 46.35] MD, -6.29 [-6.51, -6.07] MD, -6.19 [-6.45, -5.93] MD, -0.95 [-1.63, -0.27] MD, -4.12 [-5.11, -3.13]

Ye [10]	2018	Catheter slippage incidence rate Catheter infection rate Nursing satisfaction	OR, 0.14 [0.02, 1.21] OR, 0.16 [0.03, 0.84] OR, 16.47 [0.88, 308.09]

Zhang [11]	2020	Catheter slippage incidence rate Nursing satisfaction	OR, 0.09 [0.01, 0.75] OR, 17.66 [0.98, 318.99]

OR: odds ratio and MD: mean difference.

## Data Availability

The data are available from the corresponding author upon request.
